# Effect of the WeChat Platform Health Management and Refined Continuous Nursing Model on Life Quality of Patients with Acute Myocardial Infarction after PCI

**DOI:** 10.1155/2021/5034269

**Published:** 2021-11-29

**Authors:** Meifang Xu, Xiaofang Yang, Lin Liu, Yunlang Dai, Mingzhu Xu, Lin Shi

**Affiliations:** Division of Cardiology, The First Affiliated Hospital of Soochow University, Suzhou 215000, Jiangsu, China

## Abstract

The purpose was to explore the effect of the WeChat platform health management and refined continuous nursing model on life quality of patients with acute myocardial infarction (AMI) after PCI. 100 AMI patients treated in the cardiovascular medicine of the First Affiliated Hospital of Soochow University from June 2018 to June 2019 were selected as the study subjects and randomly divided into research group and reference group, with 50 cases in each group. The reference group received routine nursing after PCI, while the research group received WeChat platform health management and continuous refined nursing. There were no significant differences in sex ratio, age, BMI, complications, education level, and residence between the two groups of patients (*P* > 0.05). The MPR values of patients in the two groups after intervention were significantly higher than those before intervention (*P* < 0.05), and the MPR value in the research group after intervention was significantly higher than that in the reference group (*P* < 0.05). The SF-36 scores of patients in the two groups after intervention were significantly higher than those before intervention (*P* < 0.001), and the SF-36 score in the research group after intervention was higher than that in the reference group (*P* < 0.001). The emotional, physical, and economic dimensions of patients in the research group after intervention were significantly lower than those in the reference group (*P* < 0.001). The HAMA and HAMD scores of patients in the research group after intervention were significantly lower than those in the reference group (*P* < 0.001). The nursing satisfaction score of patients in the research group was significantly higher than that in the reference group (*P* < 0.001). The total incidence of complications of patients in the research group after intervention was significantly lower than that in the reference group (*P* < 0.05). The WeChat platform health management and refined continuous nursing model can effectively improve the medication compliance of patients after PCI, improve the life quality, alleviate depression and anxiety, and reduce postoperative complications, with a definite effect, which is worthy of promotion and application.

## 1. Introduction

In recent years, with the increasing aging population in China, the prevalence of acute myocardial infarction (AMI) is increasing year by year [1, 2]. AMI is the most serious type of coronary heart disease, and patients will suffer from pressing sensation of precordial pain and ischemic necrosis of cardiac muscle during the onset of the disease. Therefore, taking effective first-aid measures is an important means to save the lives of patients. Clinical studies have confirmed that previous medical history, dyslipidemia, smoking, obesity, emotional agitation, and so on are all risk factors for AMI [3–5]. The development and application of percutaneous coronary intervention (PCI) have significantly improved the prognosis of AMI patients, and PCI has become one of the current clinical methods for the treatment of AMI. This technique can effectively dredge the narrow or even occluded coronary artery lumen, increase myocardial blood perfusion, and effectively reduce the death risk in the acute phase of patients [6]. However, cardiovascular events may occur again in some patients after PCI, which affects the clinical treatment. The main factors are excessive anxiety or depression, low medication compliance, unhealthy lifestyles, etc. The WeChat platform is mobile software used by modern people to obtain information and communicate instantly, with the advantages of easy operation, rich content, etc. Health management by means of the WeChat platform can timely and efficiently solve the problems raised by patients, establish a good monitoring and feedback mechanism, and improve the quality of nursing service [7–9]. A refined continuous nursing model can provide good nursing services for patients discharged from hospital, help patients develop healthy life habits, and strengthen guidance and supervision of medication for patients, which is conducive to establishing a good nurse-patient relationship and improving patients' nursing satisfaction [10–12].

## 2. Materials and Methods

### 2.1. General Information

100 AMI patients treated in the cardiovascular medicine of the First Affiliated Hospital of Soochow University from June 2018 to June 2019 were selected as the study subjects and randomly divided into a research group and a reference group, with 50 cases in each group.

### 2.2. Inclusion Criteria

(1) Compliance with the clinical diagnostic criteria of AMI; (2) stable condition; and (3) good language communication or understanding ability; this study was approved by the hospital ethics committee, and the patients and their families knew the purpose and process of this experimental study and signed the informed consent.

### 2.3. Exclusion Criteria

(1) Complication with systemic coagulation disorder or malignant tumors; (2) cardiogenic shock; (3) Killip grade III-IV in AMI; and (4) the presence of mental and other cognitive disorders.

### 2.4. Methods

The reference group received routine nursing after PCI through carrying out clinical health education to patients, informing them of medication precautions, dietary intervention, psychological guidance, etc. After discharge, the patients were followed up by telephone every two weeks to inquire about medication and changes in their conditions, etc. The patients were required to have at least one outpatient follow-up every month, for 3 months. To further explore the effect of the WeChat platform health management and refined continuous nursing model on the life quality of AMI patients after PCI, 100 AMI patients treated in the cardiovascular medicine of the First Affiliated Hospital of Soochow University from June 2018 to June 2019 were selected as the study subjects, summarized and reported as follows.

The research group received the WeChat platform health management combined with refined continuous nursing model.

WeChat platform health management: during hospitalization, bed nurses set up health management records for patients meeting the requirements, including information of drugs to treat the disease, etc. A WeChat group for AMI health management was established, and patients were added into the Wechat group whose contacts were patients or family members (for elderly people who could not use smartphones). The medical staff in WeChat group included 2 doctors of cardiology, 1 cardiovascular specialist nurse, and 4–6 nurses to answer various questions after discharge and help patients make appointments for a return visit. The attending doctor gave video lectures in the group every 2 weeks to explain related knowledge of AMI disease. The patients needed to complete the tasks of clocking in, taking medicine, and measuring blood pressure and heart rate in the group every day. A reward system was formulated, and the patients could receive rewards at the end of 1 month if they performed well to encourage them to keep return visits.

Refined continuous nursing model: (1) a refined continuous nursing team was established, including department doctors and specialist nurses. The head nurses with better nursing service and rich experience served as the team leader to conduct AMI knowledge training for other team members, with the contents of nurse-patient communication skills, refined continuous nursing knowledge and specialist knowledge, etc. Records for patients were established, including name, age, contact information, home address, and medication after discharge. (2) The family visit was conducted at least once a month, and telephone follow-up was conducted at least once a week. In the visits and follow-up, the patients were told to eat more fresh fruits and vegetables, pay attention to the intake of vitamins, carbohydrates, and other nutrients, maintain a low-salt, low-oil, and low-fat diet, quit smoking and alcohol, and carry out proper physical exercise which did not cause panic or chest tightness. The patients were also guided and supervised to take antiplatelet, hypoglycemic, and antihypertensive drugs on time. Communication with family members was strengthened, and psychological counseling to patients was conducted if necessary to alleviate adverse emotions such as depression and anxiety. (3) Reminder for continuation of medication: attention was paid to the patients' medication, and telephone or short message reminders were given to patients at 4 days before the completion of medication, for 3 months.

### 2.5. Observation Indexes

Medication possession ratio (MPR) was calculated to reflect patients' medication compliance by recording the names, doses, and frequencies of drugs in the two groups. MPR = days of drug coverage/total treatment time × 100%, with a range of 0–100%. The higher the ratio was, the higher the medication compliance of the patients was.

Short-form 36 health surveys (SF-36 scoring) [13] were used to evaluate the life quality of patients in the two groups before and after intervention. There were 36 scoring items in the scale, with a total score of 100 points. The higher the score was, the higher the life quality of the patients was.

The self-perceived burden scale (SPBS) [14], a Chinese-language version, was used to evaluate the self-perceived burden of patients in the two groups after intervention. The scale consisted of 10 scoring items with a total score of 50 points. The higher the score was, the heavier the self-perceived burden of the patients was.

The Hamilton Anxiety Scale (HAMA) [15] and Hamilton Depression Scale (HAMD) [16] were used to evaluate the degree of anxiety and depression after intervention in the two groups of patients. The total score of each scale was 30 points, and the higher the score was, the more serious the anxiety or depression of the patients was.

The self-designed “Questionnaire for Patient Clinical Nursing Satisfaction” was used to evaluate the nursing satisfaction of patients in the two groups. The questionnaire was filled out at the last outpatient follow-up of the patients. There were 5 scoring items on the scale, with a total score of 100 points. The higher the score was, the higher the patients' satisfaction with the nursing was.

The incidence of clinical complications after intervention was recorded and compared between the two groups.

### 2.6. Statistical Methods

The experimental data were statistically analyzed and processed by SPSS21.0 software. GraphPad Prism 6 (GraphPad Software, San Diego, USA) was used to draw pictures of the data. The count data were tested by x^2^, expressed by [n (%)], and the measurement data were measured by the *t*-test, expressed by ($\bar{x}\pm s$). The difference was statistically significant when *P* < 0.05.

## 3. Results

### 3.1. Comparison of Clinical Data between the Two Groups of Patients

There were no significant differences in sex ratio, age, BMI, complications, education level, and residence between the two groups of patients (*P* > 0.05), which were comparable, as shown in Table 1.

### 3.2. Comparison of MPR Values between the Two Groups of Patients before and after Intervention

The MPR values of patients in the two groups after intervention were significantly higher than those before intervention (*P* < 0.05), and MPR value in the research group after intervention was significantly higher than that in the reference group (*P* < 0.05), as shown in Figure 1.

### 3.3. Comparison of SF-36 Scores between the Two Groups of Patients before and after Intervention

The SF-36 scores of patients in the two groups after intervention were significantly higher than those before intervention (*P* < 0.05), and the SF-36 score of patients in the research group after intervention was significantly higher than that in the reference group (*P* < 0.05), as shown in Figure 2.

### 3.4. Comparison of SPBS Scores between the Two Groups of Patients after Intervention

The emotional, physical, and economic dimensions of patients in the research group after intervention were significantly lower than those in the reference group (*P* < 0.05), as shown in Table 2.

### 3.5. Comparison of HAMA and HAMD Scores between the Two Groups of Patients after Intervention

The HAMA and HAMD scores of patients in the research group after intervention were significantly lower than those in the reference group (*P* < 0.05), as shown in Table 3.

### 3.6. Comparison of Nursing Satisfaction Scores between the Two Groups of Patients

The nursing satisfaction score of patients in the research group was significantly higher than that in the control group (*P* < 0.05), as shown in Figure 3.

### 3.7. Comparison of Complications between the Two Groups of Patients after Intervention

The total incidence of complications after intervention in the research group was significantly lower than that in the reference group (*P* < 0.05), as shown in Table 4.

## 4. Discussion

As a common clinical cardiovascular disease, AMI refers to acute myocardial necrosis caused by severe and lasting myocardial ischemia [17]. With the increasing improvement of the PCI technique, this technique has gradually become the first treatment method to achieve reperfusion of infarct-related vessels and restore normal myocardial function in AMI patients. Clinical studies have confirmed that PCI has a significant short-term clinical efficacy in AMI patients, but cardiovascular events are likely to occur again with the changes in patients' lifestyles after discharge. Besides, the patients have anxiety, depression, and other adverse emotions and worry about the cost of treatment, which seriously affects the disease treatment and prognosis. Routine nursing service after PCI confines the focus of nursing to patients during hospitalization, implements clinical health education for patients about to be discharged, and informs patients of basic nursing services such as medication methods and dosage, which results in a “disruption” state after patients are discharged from hospital. For patients with low knowledge of their own diseases or more negative emotions, their medication compliance after discharge is worse [18–20].

WeChat, as a common communication tool for young and middle-aged people, can make up for the deficiencies of clinical nursing in hospitals to some extent and break the limitation of routine nursing after PCI, which truly provides more high-quality services for patients. Chapman et al. [21] believe that WeChat, as a real-time communication tool, can help doctors timely understand the condition and psychological changes of discharged patients and take effective measures to address their situation to break the limitations of space and time and meet the nursing needs of patients after discharge. In this study, WeChat platform health management was implemented for patients after PCI, urging patients to clock in the group every day and report medication. The MPR value of patients after intervention was significantly higher than that of the reference group (*P* < 0.001). Nicole R. Pinelli et al. [20] pointed out in their paper that, “after the implementation of WeChat platform health management for rectal cancer patients undergoing radical resection, the MPR value of patients after intervention was (85.67 ± 3.28)%, significantly higher than that of the reference group (75.21 ± 3.32)%,” indicating that WeChat platform health management can effectively improve the treatment compliance of discharged patients and accelerate physical rehabilitation. In addition, the refined continuous nursing model provides comprehensive, continuous, and refined nursing services for discharged patients, which focuses on solving all kinds of problems of patients at home, supervises medication on time, strengthens communication with patients, timely alleviates negative emotions of patients, and maintains good nurse-patient relationship [22, 23].

## 5. Conclusions

How to improve the medication compliance, improve the life quality, and reduce cardiovascular complications of patients after PCI has become a hot topic in the medical field [24–26]. The long rehabilitation process of AMI and a variety of oral drugs for a long time in the treatment result in poor treatment compliance. This study showed that the HAMA and HAMD scores of patients after refined continuous nursing were significantly lower than those of the reference group (*P* < 0.001), indicating that this nursing model can effectively alleviate the adverse emotions of patients after PCI and is beneficial to treatment.

However, this study also had some shortcomings. Single cases were selected, and the results of the study were easily affected by regions. Besides, the duration of continuous nursing was only 3 months, and there was a lack of long-term follow-up studies for patients after PCI. It is suggested that the selection of samples should follow the diversification principle and the postoperative nursing service time should be prolonged.

In summary, the WeChat platform health management combined with refined continuous nursing model can significantly improve the medication compliance of patients after PCI, alleviate their negative emotions, improve the life quality, and reduce their self-perceived burden, with high safety, which is worthy of application and promotion.

## Figures and Tables

**Figure 1:** Comparison of MPR values between the two groups of patients before and after intervention ($\bar{x}\pm s$). *Note.* The abscissa represents before intervention and after intervention, and the ordinate represents MPR value (%). The MPR values of the research group were (73.29 ± 8.45)% and (86.25 ± 8.03)%, respectively, before and after intervention. The MPR values of the reference group were (73.32 ± 8.42)% and (77.43 ± 8.06)%, respectively, before and after intervention. ^*∗*^ indicates that there was a significant difference in MPR values in the research group before and after intervention (*t* = 7.862, *P*=0.000); ^*∗∗*^ indicates that there was a significant difference in MPR values in the reference group before and after intervention (*t* = 2.493, *P*=0.014); and ^*∗∗∗*^ indicates that there was a significant difference in MPR values between the two groups after intervention (*t* = 5.482, *P*=0.000).

**Figure 2:** Comparison of SF-36 scores between the two groups of patients before and after intervention ($\bar{x}\pm s$). *Note*. The abscissa represents before intervention and after intervention, and the ordinate represents SF-36 scores (points). The SF-36 scores of the research group were (54.27 ± 6.35)% and (74.26 ± 6.44)%, respectively, before and after intervention. The SF-36 scores of the reference group were (54.30 ± 6.32)% and (63.84 ± 6.36)%, respectively, before and after intervention. ^*∗*^ indicates that there was a significant difference in SF-36 scores in the research group before and after intervention (*t* = 15.629, *P*=0.000); ^*∗∗*^ indicates that there was a significant difference in SF-36 scores in the reference group before and after intervention (*t* = 7.524, *P*=0.000); and ^*∗∗∗*^ indicates that there was a significant difference in SF-36 scores between the two groups after intervention (*t* = 8.140, *P*=0.000).

**Figure 3:** Comparison of nursing satisfaction scores between two groups of patients ($\bar{x}\pm s$). *Note*. The abscissa represents the research group and reference group, respectively, and the ordinate represents the nursing satisfaction score. The nursing satisfaction score of patients was (87.68 ± 4.82) points in the research group and (72.17 ± 4.76) points in the reference group. ^*∗*^ indicates that there was a significant difference in nursing satisfaction scores between the two groups of patients (*t* = 16.190, *P*=0.000).

**Table 1:** Comparison of clinical data between the two groups of patients.

Category	Research group (*n* = 50)	Reference group (*n* = 50)	*x* ^2^/*t*		*P*
Gender			0.271		0.603
Male	40 (80.00%)	42 (84.00%)			
Female	10 (20.00%)	8 (16.00%)			
Average age (years)	56.27 ± 24.53	56.29 ± 24.57	0.004		0.997
BMI (kg/m^2^)	21.34 ± 1.02	21.36 ± 1.04	0.097		0.923
Complications			0.178		0.673
Hypertension	32 (64.00%)	34 (68.00%)			
Diabetes mellitus	18 (36.00%)	16 (32.00%)			
Education level					
College and above	12 (24.00%)	14 (28.00%)	0.208		0.648
High school	15 (30.00%)	17 (34.00%)	0.184		0.668
Middle school and below	23 (46.00%)	19 (38.00%)	0.657		0.418
Residence (cases)			0.045		0.832
City	34 (68.00%)	33 (66.00%)			
Country	16 (32.00%)	17 (34.00%)			

**Table 2:** Comparison of SPBS scores between the two groups of patients before and after intervention ($\bar{x}\pm s$, points).

Group	*n*	Emotional dimension	Physical dimension	Economic dimension
Research group	50	24.18 ± 3.46	21.26 ± 4.32	17.24 ± 2.63
Reference group	50	31.22 ± 3.27	29.31 ± 4.36	22.31 ± 2.84
*t*		10.456	9.274	9.262
*P*		0.000	0.000	0.000

**Table 3:** Comparison of HAMA and HAMD scores between the two groups after intervention ($\bar{x}\pm s$, points).

Group	*n*	HAMA	HAMD
Research group	50	16.45 ± 3.36	14.38 ± 3.41
Reference group	50	21.52 ± 3.28	18.62 ± 3.27
*t*		7.635	6.346
*P*		0.000	0.000

**Table 4:** Comparison of complications between the two groups of patients after intervention [n (%)].

Group	*n*	Arrhythmia	Thrombocytopenia	Angina pectoris	Total incidence
Research group	50	1 (2.00%)	2 (4.00%)	0 (0.00%)	6.00％ (3/50)
Reference group	50	3 (6.00%)	4 (8.00%)	3 (6.00%)	20.00％ (10/50)
*X* ^2^					4.332
*P*					0.037

## Data Availability

The datasets used and/or analyzed during the current study are available from the corresponding author on reasonable request.
